The article "14‐3‐3ζ promotes gliomas cells invasion by regulating Snail through the PI3K/AKT signaling" was retracted in 2023. Reasons: errors in the data; errors in the images; duplicated images; unreliable results or conclusions.

# 14‐3‐3ζ promotes gliomas cells invasion by regulating Snail through the PI3K/AKT signaling

**DOI:** 10.1002/cam4.1950

**Published:** 2019-01-18

**Authors:** Junjun Li, Hao Xu, Qiangping Wang, Sihua Wang, Nanxiang Xiong

**Affiliations:** ^1^ Department of Neurosurgery Union Hospital Tongji Medical College Huazhong University of Science and Technology Wuhan China; ^2^ Department of Thoracic surgery Union Hospital Tongji Medical College Huazhong University of Science and Technology Wuhan China

**Keywords:** 14‐3‐3ζ, gliomas, invasion, PI3K/AKT, Snail

## Abstract

14‐3‐3ζ has been reported to function as critical regulators of diverse cellular responses. However, the role of 14‐3‐3ζ in gliomas progression remains largely unknown. The expression level of 14‐3‐3ζ and Snail was detected by Western blot analysis and quantitative polymerase chain reaction in different grades of human gliomas. The effect of 14‐3‐3ζ on gliomas progression was measured using cell migration and invasion assay, the colony formation experiment, and CCK‐8 assay. The effect of 14‐3‐3ζ on PI3K/AKT/Snail signaling protein expression levels was tested by Western blotting. Firstly, 14‐3‐3ζ was often up‐regulated in high‐grade gliomas relative to low‐grade gliomas, and this overexpression was significantly related to tumor size, Karnofsky Performance Scale score and weaker disease‐free survival. Secondly, the overexpression of 14‐3‐3ζ promoted gliomas cells proliferation, migration, and invasion. Conversely, the knockdown of 14‐3‐3ζ suppressed gliomas cells proliferation, migration, and invasion. Furthermore, subsequent mechanistic studies showed that 14‐3‐3ζ could activate PI3K/AKT **/**Snail signaling pathway to facilitate gliomas cells proliferation, migration, and invasion. This study shows that the overexpression of 14‐3‐3ζ can promote remarkably gliomas cells proliferation, migration, and invasion by regulating the Snail protein expression through activating PI3K/AKT signaling, and it may serve as a potential prognostic marker and therapeutic target for gliomas.

## 1 INTRODUCTION

Gliomas are the most common primary and lethal tumors coming from the central nervous system.^1^ According to the World Health Organization classification, they are graded from I to IV on the basis of their degree of malignancy.^2^ Despite modern multimodal therapy, including surgical resection as well as adjuvant radiation and chemotherapy therapy, the conditions of prognosis are still not optimistic.^3^

The 14‐3‐3 proteins compose a family of highly conserved proteins found in all eukaryotic organisms.^4^ These 29‐31 kDa acidic proteins are combined with phosphorylated serine/threonine in the target proteins.^5^3‐3 proteins have not any catalytic activity; however, they exert their effect on regulating catalytic activity of target proteins or sub‐cellular localization and on mediating formation of protein complexes.^6^3‐3 proteins communicate with many proteins that potentially modulate a diverse number of cellular processes.^7^, ^8^, ^9^ Therefore, 14‐3‐3 proteins potentially modulate multiple pathways involved in diverse biological functions and tumor progression. In humans, there are seven differently identified subtypes (ζ, σ, β, ε, η, γ, θ),^10^ which were initially described as enzyme cofactors affecting the activity of protein kinase C and Raf‐1.^11^ Accumulating evidences have shown that the 14‐3‐3 family is related to the product of oncogene. 14‐3‐3ζ is a member of the 14‐3‐3 family broadly known for its role in promoting the development and progression of human cancers. 14‐3‐3ζ is one of the central proteins induced by TGF‐β, which can promote the epithelial‐mesenchymal transition in cancer cells.^12^ In addition, 14‐3‐3ζ can combine with the tumor suppressor tuberin to deter the phosphoinositide‐3′‐kinase signaling downstream of AKT.^13^

14‐3‐3ζ proteins have also been proved to intercommunicate with other survival‐promoting proteins such as phosphoinositide 3‐kinase (PI3K) and growth factor receptors.^14^ However, the mechanism of those interactions, especially related to tumor progression, is not well understood.^15^, ^16^ In this study, we demonstrate that 14‐3‐3ζ overexpression is related to the malignancy of gliomas, and Snail is up‐regulated by 14‐3‐3ζ through activating PI3K/AKT signaling.

The article "14‐3‐3ζ promotes gliomas cells invasion by regulating Snail through the PI3K/AKT signaling" was retracted in 2023. Reasons: errors in the data; errors in the images; duplicated images; unreliable results or conclusions.

## 2 METHODS

### 2.1 Bioinformatics database

The GBM gene expression came from The Cancer Genome Atlas (http://cancergenome.nih.gov). Data processing used cBioPortal (http://cbioportal.org) and GraphPad Prism 5 Software (GraphPad Prism Software Inc, San Diego, CA, USA).

### 2.2 Cell lines and reagents

U‐87 and U‐251 cells (American Type Culture Collection, Manassas, VA, USA) were cultured in a DMEM medium (Hyclone, Logan County, KY, USA) containing 10% fetal bovine serum (Gibco, Grand Island, NE, USA) and 1% of 100 U/L penicillin and 100 mg/L streptomycin (Gibco). BEZ235 (2‐methyl‐2‐(4‐(3‐methyl‐2‐oxo‐8‐(quinolin‐3‐yl)‐2,3‐dihydroimidazo[4,5‐c]quinolin‐1‐yl)phenyl)propanenitrile, Sigma‐Aldrich, Kansas City, MO, USA) and LY294002 (2‐morpholino‐8‐phenyl‐4H‐chromen‐4‐one; Sigma‐Aldrich) were purchased from Sigma‐Aldrich. Anti‐14‐3‐3 zeta (ab51129) antibodies and Anti‐Snail (ab53519) antibodies were purchased from Abcam (Cambridge, MA, USA); Anti‐PI3K p85 (4257), Anti‐P‐PI3K p85 (4292), anti‐AKT (4691), anti‐P‐AKT (Ser473) (4060), and anti‐β‐actin(4970) antibodies were bought from Cell Signaling Technology (Danvers, MA, USA).

The article "14‐3‐3ζ promotes gliomas cells invasion by regulating Snail through the PI3K/AKT signaling" was retracted in 2023. Reasons: errors in the data; errors in the images; duplicated images; unreliable results or conclusions.

### 2.3 Patients

Tumor samples collected from patients during a neurosurgical resected gliomas were immediately frozen and kept at −80°C. All patients received their informed consent for the neurosurgical procedures and for anonymous scientific analysis of pathological tissue according to the guidelines of the Human Research Committee of Huazhong University of Science and Technology and China Anti‐Cancer Association (CACA).

### 2.4 Plasmid constructs and transfection

Lentiviruses containing shRNAs targeting 14‐3‐3ζ and Snail were purchased from Shandong ViGene (ViGene, Shandong, China) and used to infect cells. The 14‐3‐3ζ target sequence was 5′‐GCAATTACTGAGAGACAACTT‐3′, and the Snail target sequence was 5′‐GCTGAGCTGTTACTAGGACAA‐3′. The short hairpin RNAs were designed, based on the 14‐3‐3ζ sequence: 5′‐GACAAGGTCATCTCCTACAAT‐3′. Cells infected with empty vector or scrambled shRNA were acted as controls.

### 2.5 Cell migration and invasion assays

Cell invasion and migration experiments were performed using a transwell system (Corning, NY) on the basis of the manufacturer's protocol. To evaluate the invasion ability, filters were precoated with Matrigel (BD Biosciences, Becton, Dickinson and Company, Jersey city, NJ, USA). Approximately 1 × 10^4^ cells in serum‐free DMEM were added to the top chamber, and the bottom chamber was full of DMEM containing 20% FBS. After incubation for 24 hours, the cells on the upper surface were softly removed with cotton swab, and then the membrane was fixed in 4% methanol for 15 minutes and stained with 0.1% crystal violet solution for 30 minutes. The cells that migrated to the down surface of the membrane were captured, and the cell number was counted under a microscope. The same experimental design was adopted for migration assays excepting that the filters were not precoated with Matrigel.

### 2.6 Cell counting Kit‐8 (CCK‐8) assay

The cells were resuspended at the logarithmic growth phase and then cultured incomplete culture medium. The cell density was adjusted into 5 × 10^3^/well in 96‐well plates. After the cells were incubated adherent to wall for 24 hours, the cells culture medium was discarded. Then treatment with CCK‐8 (10 μL) according to the manufacturer's protocol, the absorbance was detected using a microplate reader at 450 nm wavelength with subtraction of the baseline reading.

### 2.7 Colony formation assay

For each cell line, 600 cells were plated in triplicate into 6‐well plates containing 3 mL of culture medium with 20% FBS. Cells were cultivated for 2 weeks at 37°C and 5% CO_2_, during which period the culture medium was not changed. Then cells were fixed with 4% formaldehyde and stained with crystal violet. The colonies with a diameter exceeding 2 mm were counted and photographed. Triplicate experiments were performed.

The article "14‐3‐3ζ promotes gliomas cells invasion by regulating Snail through the PI3K/AKT signaling" was retracted in 2023. Reasons: errors in the data; errors in the images; duplicated images; unreliable results or conclusions.

### 2.8 Western blot analysis

Cells were lysed and equal amounts of protein lysates were electrophoresed in a 12% SDS‐PAGE gel at 120 V for 2 hours and transferred to a PVDF membrane (Millipore). The membrane was incubated with 5% fat‐free milk intris‐buffered saline tween‐20(TBST) for 2 hours. Then, the membranes were hatched and probed with primary and secondary antibodies, and the bound antibodies were detected with the Pierce ECL (BOSTER, Wuhan, China) and exposed to X‐ray film. The analysis of band densities was adopted using Image J software (Bethesda, MA, USA).

### 2.9 qRT‐PCR

Total RNA was extracted from gliomas samples using TRIZOL reagent (Thermo Fisher Scientific, Carisbad, CA, USA). Reverse Transcription and quantitative PCR was performed with using the SYBR. Premix Ex Taq™ Kit (Takara, Tokyo, Japan). The sequences of the 14‐3‐3ζ primers were as follows: forward, 5′‐TGATCCCCAAAATGCTTCACAAG‐3′; reverse, 5′‐GCCAAGTAACGGTAGTAATCTCC ‐3′. The sequences of the Snail primers were as follows: forward, 5′‐TCGGAAGCCTAACTACAGCGA‐3′; reverse, 5′‐ AGATGAGCATTGGCAGCGAG ‐3′. The sequences of the GAPDH primers were as follows: forward, 5′‐GGAGCGAGATCCCTCCAAAAT‐3′; reverse, 5′‐GGCTGTTGTCATACTTCTCATGG‐3′. GAPDH was acted as a control for normalizing the gene expression of 14‐3‐3ζ. Three independent experiments were repeated. The obtained data were calculated by 2^−ΔΔCt^ and evaluated for statistical analysis followed by an unpaired sample *t* test.

### 2.10 Immunohistochemical and immunofluorescence staining analyses

Tissue sections were fixed with 4% paraformaldehyde and then permeabilized with 0.5% Triton X‐100, washed thrice with PBS, and incubated in blocking buffer (5% bovine serum albumin) for 1 hour. Antibodies were suspended in blocking buffer and incubated overnight. U‐87 and U‐251 cells were incubated with Cy3‐conjugated rabbit or mouse secondary antibodies (1:100; Promoter, Wuhan, China), counterstained with 4′, 6‐diamidino‐2‐phenylindole (DAPI), and then mounted with anti‐fade solution (Molecular Probes, Eugene, CA, USA). The fluorescence was visualized with an Olympus FV500 laser scanning confocal microscope (Olympus America, Inc.) and processed using Metamorph 2D deconvolution software (Molecular Devices Co., Oakland, CA, USA).

Slides (4 μm) of formalin‐fixed and paraffin‐embedded tissue sections were incubated with 14‐3‐3ζ antibody (1:100) and subsequently incubated with Cy3‐conjugated goat anti‐rabbit antibody (Promoter) at a concentration of 1:100 for 30 minutes at 37°C.

The article "14‐3‐3ζ promotes gliomas cells invasion by regulating Snail through the PI3K/AKT signaling" was retracted in 2023. Reasons: errors in the data; errors in the images; duplicated images; unreliable results or conclusions.

The immunohistochemically semiquantitative scoring system based on staining intensity and distribution adopting the immunoreactive score (IRS) was applied as described 17 and as following (IRS = SI [staining intensity] × PP [percentage of positive cells]). SI was determined as following (0 = negative; 1 = weak; 2 = moderate; and 3 = strong). PP was defined as following (0, <1%; 1, 1%‐10%; 2, 11%‐50%; 3, 51%‐80%; and 4, >80% positive cells), leading to scores from 0 to 12. Ten visual fields coming from different areas of each sample were adopted for the IRS evaluation.

### 2.11 Statistical analysis

The Empower Stats statistical software program version 2.16.1 (San Diego, CA, USA) was adopted to perform the statistical analysis. The mRNA levels of 14‐3‐3ζ and Snail in gliomas samples in different grades of human gliomas were compared using a paired Student *t* test. Clinical correlations were analyzed by two‐tailed Student's *t* tests. The log‐rank tests and Kaplan‐Meier plots were used to perform the survival analyses. The Cox regression model was used to perform the multivariate survival analyses.

## 3 RESULTS

### 3.1 The 14‐3‐3ζ expression of bioinformatics analysis and it is often overexpressed in human gliomas

The genome sequence of 20 samples of normal brain tissue and 36 glioblastoma tissues was adopted from glioblastoma whole gene expression map database of the Cancer and Tumor Gene Mapping (TCGA) Plan Database. We found that the expression of 14‐3‐3ζ in the tumors was significantly higher than that in normal brains by the analysis of bioinformatics data (Figure 1A, *P* < 0.001). The expression of 14‐3‐3ζ was measured by RT‐PCR in different grades of human gliomas. A significant difference in 14‐3‐3ζ gene expression was obviously observed in different grades of human gliomas (Figure 1B, *P* < 0.01). Sixteen gliomas tissues were assessed for 14‐3‐3ζ expression by Western blot, including four grade I, four grade II, four grade III, and four grade IV. Western blot analysis showed that 14‐3‐3ζ was often exhibiting higher expression at a higher grade (Figure 1C). Then we performed immunohistochemical analyses to detect the expression level of 14‐3‐3ζ in 49 human gliomas specimens. As shown in Figure 1D, the immune staining intensity of 14‐3‐3ζ was significantly different in different grades of human gliomas. Quantification analyses further demonstrated that 14‐3‐3ζ protein expression was obviously increased (Figure 1E, *P* < 0.01). The correlation of 14‐3‐3ζ expression with clinic pathological features in 49 gliomas samples with informative IHC was statistically analyzed. The results indicated that the increase in 14‐3‐3ζ expression was vitally related to Karnofsky Performance Scale (KPS) score (*P* = 0.005) and recurrence (*P* = 0.009, Table 1), which was accord with KPS as independent predictors for survival.^18^ As shown in Table 2, high expression of 14‐3‐3ζ was related to a significantly increased risk of tumor recurrence in gliomas patients (*P* < 0.001) compared to those with low 14‐3‐3ζ expression by univariate Cox regression analyses (Table 2). Multivariate Cox regression analysis indicated that 14‐3‐3ζ could predict poor survival when 14‐3‐3ζ expression (*P *<* *0.001), tumor grade (*P *<* *0.001) and tumor recurrence were included (*P *<* *0.001; Table 2). These results demonstrate a significant correlation of the expression of 14‐3‐3ζ with the prognosis of gliomas. Besides, Kaplan‐Meier analysis indicated that the increase in 14‐3‐3ζ expression was vitally related to weaker disease‐free survival (DFS) rates in gliomas patients (Figure 1F, *P* = 0.003). Multivariate Cox regression analysis showed that, compared with tumors containing high 14‐3‐3ζ expression, the hazard ratio (HR) for DFS with tumors containing low 14‐3‐3ζ expression was higher (HR 1.63 95% CI 1.09‐2.17, *P* = 0.003).

The article "14‐3‐3ζ promotes gliomas cells invasion by regulating Snail through the PI3K/AKT signaling" was retracted in 2023. Reasons: errors in the data; errors in the images; duplicated images; unreliable results or conclusions.

**Figure 1:** 14‐3‐3ζ is often overexpressed in human gliomas. A, The expression of 14‐3‐3ζ in TCGA glioblastoma databases. B, Relative expression levels of 14‐3‐3ζ detected by RT‐PCR in 49 pairs of gliomas specimens. C, Western blot test of 14‐3‐3ζ expression in total frozen samples lysates deriving from 16 different grades of human gliomas specimens. D, Representative immunohistochemical staining of 14‐3‐3ζ expression in different grades of human gliomas specimens. Bars: 200/100 μm. (original magnification, 100× and 200×). E, 14‐3‐3ζ expression scores are depicted as dot blots. Different grades of gliomas specimens were compared using paired Student's *t* test. n = 49. F, Kaplan‐Meier analysis demonstrating the relevance between poorer disease‐free survival rates and the decrease in 14‐3‐3ζ expression of gliomas patients. *P <* *0.05, **P <* *0.01, ***P <* *0.001

**Table 1:** Association of 14‐3‐3ζ expression with clinicopathological characteristics in human gliomas

Features	No.	14‐3‐3ζ		*P*‐value
		Low	High	
Age (years)				
<50	26	15	11	0.39
≥50	23	16	7	
Gender				
Male	27	14	13	0.07
Female	22	17	5	
Tumor size, cm				
<5	28	22	6	0.01*
≥5	21	9	12	
Tumor location				
Supratentorial	35	23	12	0.57
Subtentorial	14	8	6	
Karnofsky performance scale				
<90	26^a^	12^a^	14^a^	0.005**
≥90	21	18	3	
WHO grade				
Low‐grade(I + II)	31	24	7	0.007**
High‐grade(III + IV)	18	7	11	
Tumor recurrence				
No	33	25	8	0.009**
Yes	16	6	10	

*P < 0.05; **P < 0.01.

a Partial data not available; statistics based on available data.

The article "14‐3‐3ζ promotes gliomas cells invasion by regulating Snail through the PI3K/AKT signaling" was retracted in 2023. Reasons: errors in the data; errors in the images; duplicated images; unreliable results or conclusions.

**Table 2:** Univariate and multivariate analyses of various prognostic parameters in patients with gliomas Coxregression analysis

	Univariate analysis			Multivariate analysis		
	*P* value	Hazard ratio	95% confidence interval	*P* value	Hazard ratio	95% confidence interval
14‐3‐3ζ	<0.001	2.569	1.950‐4.342	<0.001	1.933	1.693‐3.317
Tumor size, cm	0.023	1.265	1.189‐2.421	<0.001	2.537	1.685‐3.983
Karnofsky performance scale	<0.001	1.576	1.243‐1.909	0.008	1.447	1.253‐1.812
WHO grade	<0.001	2.651	1.476‐3.285	<0.001	1.553	1.216‐2.869
Tumor recurrence	<0.001	1.764	1.216‐2.895	<0.001	1.475	1.284‐3.218

### 3.2 Overexpression of 14‐3‐3ζ promotes gliomas cells proliferation, migration, and invasion

Because 14‐3‐3ζ overexpression was associated with gliomas tumor size and recurrence, the role of 14‐3‐3ζ in tumor cells proliferation, migration, and invasion was researched. U‐87 and U‐251 cells were stably transfected with the Lentiviruses containing sh14‐3‐3ζ, and the expression of the 14‐3‐3ζ was measured by qRT‐PCR and Western blotting (Figure 2A,B). We thus used the CCK‐8 assay, colony formation assay, and transwell assay to test the effect of 14‐3‐3ζ on the proliferation, migration, and invasion potential of the gliomas cells. The results indicated that 14‐3‐3ζ overexpression promoted gliomas cells proliferation, migration, and invasion significantly (Figure 2C‐F).

**Figure 2:** Overexpression of 14‐3‐3ζ promotes gliomas cells proliferation, migration, and invasion. A and B, Validation of shRNA against 14‐3‐3ζ in U‐87 and U‐251 cells by qRT‐PCR and Western blotting. C, Growth curves between 14‐3‐3ζ‐shRNA and scramble control‐infected cells by CCK‐8 assay. The results are demonstrated as the mean ± SD of seven independent experiments. D, Overexpression of 14‐3‐3ζ importantly increased colony formation in U‐87 and U‐251 cells. Quantitative data for colony numbers are expressed in the right panel. E and F, Transwell migration and invasion assay showing that overexpression of 14‐3‐3ζ promoted cell migration and invasion. The numbers of migrating and invading cells are summarized in the right panel. The results are expressed as the mean ± SD of five independent experiments. Bars: 400 μm. *P <* *0.05, **P <* *0.01. none, Noninfected cells

### 3.3 Knockdown of 14‐3‐3ζ suppresses gliomas cells proliferation, migration, and invasion

Then we knocked down 14‐3‐3ζ with the short hairpin RNAs in gliomas cells U‐87 and U‐251. The transfection efficiency was verified with qRT‐PCR and Western blotting (Figure 3A,B); we thus used the CCK‐8 assay, colony formation assay, and transwell assay to test the effect of 14‐3‐3ζ on the proliferation, migration, and invasion potential of the gliomas cells. The results indicated that 14‐3‐3ζ silencing inhibited gliomas cells proliferation, migration, and invasion significantly (Figure 3C‐F).

The article "14‐3‐3ζ promotes gliomas cells invasion by regulating Snail through the PI3K/AKT signaling" was retracted in 2023. Reasons: errors in the data; errors in the images; duplicated images; unreliable results or conclusions.

**Figure 3:** Knockdown of 14‐3‐3ζ inhibits gliomas cells proliferation, migration, and invasion. A and B, Validation of siRNA against 14‐3‐3ζ in U‐87 and U‐251 cells by qRT‐PCR and Western blotting. C, Growth curves between 14‐3‐3ζ‐siRNA and scramble control‐infected cells by CCK‐8 assay. The results are demonstrated as the mean ± SD of seven independent experiments. D, Knockdown of 14‐3‐3ζ importantly inhibited colony formation in U‐87 and U‐251 cells. Quantitative data for colony numbers are expressed in the right panel. E and F, Transwell migration and invasion assay showing that knockdown of 14‐3‐3ζ inhibited cell migration and invasion. The numbers of migrating and invading cells are summarized in the right panel. The results are expressed as the mean ± SD of five independent experiments. Bars: 400 μm. *P <* *0.05, **P <* *0.01. none, Noninfected cells

### 3.4 Snail is involved in 14‐3‐3ζ‐regulated gliomas cells proliferation, migration, and invasion

It has been reported that Snail proteins involve in a variety of cellular processes through a number of different mechanisms.^19^ Previous studies have reported that overexpression of the Snail could facilitate the proliferation and invasion of gliomas cells.^20^ Therefore, we supposed that up‐regulation of 14‐3‐3ζ might promote Snail activation or expression, thereby inducing the increase of gliomas cells proliferation and invasion. Then we knocked down 14‐3‐3ζ with the short hairpin RNAs in gliomas cells U‐87 and U‐251 and found that, compared with the control group, the protein level of p‐PI3K, p‐AKT, and Snail markedly decreased (Figure 4A). Besides, to test the correlation between the protein level of 14‐3‐3ζ and Snail, we measured their expression level in 49 gliomas samples with using qRT‐PCR (Figure 4B). To test whether Snail is involved in 14‐3‐3ζ‐regulated gliomas cells proliferation and invasion, we overexpressed Snail with using Lentiviruses containing shRNAs targeting Snail in U‐87 and U‐251 cells (Figure 4C). Snail overexpression rescued the effects of 14‐3‐3ζ silencing on inhibiting U‐87 and U‐251 cell proliferation (Figure 4D), colony formation (Figure 4E), migration (Figure 4F), and invasion (Figure 4G). These results indicate that 14‐3‐3ζ promotes the migration and invasion of gliomas cells by regulating Snail protein expression.

**Figure 4:** Snail is involved in 14‐3‐3ζ‐regulated gliomas cells proliferation, migration, and invasion. A, Knockdown of 14‐3‐3ζ decreased the protein level of p‐PI3K, p‐AKT, and Snail. B, The protein level between 14‐3‐3ζ and Snail showed the positive correlation in 49 gliomas samples with using qRT‐PCR. C, Validation of shRNA against Snail in U‐87 and U‐251 cells by Western blotting. D, Growth curves were performed by CCK‐8 assay. The results are showed as the mean ± SD of seven independent experiments. E, Overexpression of Snail rescued the effects of knockdown of 14‐3‐3ζ in inhibiting U‐87 and U‐251 cell colony formation. E and F, Transwell migration and invasion experiment were performed as described in the Methods. The numbers of migrating and invading cells are summarized in the right panel. The results are expressed as the mean ± SD of five independent experiments. Bars: 400 μm. *P <* *0.05, **P <* *0.01. none, Noninfected cells

The article "14‐3‐3ζ promotes gliomas cells invasion by regulating Snail through the PI3K/AKT signaling" was retracted in 2023. Reasons: errors in the data; errors in the images; duplicated images; unreliable results or conclusions.

### 3.5 14‐3‐3ζ overexpression increases Snail through PI3K/AKT signaling

PI3K/AKT signaling involves in a series of cellular processes through different mechanisms.^21^ However, it is unclear whether these processes are involved in 14‐3‐3ζ‐mediated Snail protein expression. Therefore, we surmised whether 14‐3‐3ζ up‐regulation increased Snail protein level by PI3K/AKT signaling pathway. To validate the hypothesis, we cocultured 14‐3‐3ζ‐overexpressing cells with two chemical inhibitors of PI3K/AKT signaling pathway, such as BEZ235 and LY294002. At first, their inhibition efficiency in U‐87 and U‐251 cells was verified by p85 (Figure 5A). The p‐AKT^ser473^ protein expression level following 14‐3‐3ζ‐overexpressing in U‐87 and U‐251 cells was attenuated by BEZ235 and LY294002 (Figure 5B). Next, the Snail protein expression level following 14‐3‐3ζ‐overexpressing in U‐87 and U‐251 cells was also attenuated by BEZ235 and LY294002 (Figure 5C). All of these results strongly indicate that 14‐3‐3ζ‐overexpressing increases Snail protein expression level through PI3K/AKT signaling pathway.

**Figure 5:** 14‐3‐3ζ overexpression increases Snail through PI3K/AKT signaling. A, U‐87 and U‐251 cells transfected with 14‐3‐3ζ plasmid and cultured with PI3K/AKT signaling inhibitors were reaped, and the lysates were immunoblotted for P‐p85, Tot.p85, and β‐actin. B, U‐87 and U‐251 cells transfected with 14‐3‐3ζ plasmid and cultured with PI3K/AKT signaling inhibitors were reaped, and the lysates were immunoblotted for p‐AKT^S^ ^er473^, AKT, and β‐actin. C, U‐87 and U‐251 cells transfected with 14‐3‐3ζ plasmid and cultured with PI3K/AKT signaling inhibitors were reaped, and the lysates were immunoblotted for Snail, Slug, and β‐actin. *P < 0.05

### 3.6 The silence of 14‐3‐3ζ suppresses the tumorigenesis in vivo

We then investigated whether 14‐3‐3ζ silencing suppressed the tumor growth of gliomas cells in vivo. Thus, the cell lines that stably overexpressed Snail and silenced 14‐3‐3ζ in U‐87 and U‐251 were constructed and injected into nude mice through the subcutaneous injection. After about 6 weeks, the mice were sacrificed, and the subcutaneous tumors were extracted and weighed (Figure 6A,B,S1 and S2). Immunofluorescence staining of Ki‐67 of the subcutaneous tumors showed that, compared with the control group, 14‐3‐3ζ silencing suppressed the expression of Ki‐67. However, Snail overexpression rescued the effects of 14‐3‐3ζ silencing on inhibiting the expression of Ki‐67 (Figure 6C). All of these results strongly indicate that 14‐3‐3ζ silencing could suppress the tumorigenesis in vivo.

The article "14‐3‐3ζ promotes gliomas cells invasion by regulating Snail through the PI3K/AKT signaling" was retracted in 2023. Reasons: errors in the data; errors in the images; duplicated images; unreliable results or conclusions.

**Figure 6:** Knockdown of 14‐3‐3ζ suppressed the tumorigenesis in *vivo*. A and B, Images of the xenografted tumors of nude mice of injecting the infected U‐87 and U‐251 cells. The down panel shows the volumes and weights of tumors. There were three mice in each group. *P <* *0.05, **P <* *0.01. none, Noninfected cells. C, Immunofluorescence staining of Ki‐67 of the subcutaneous tumors of different group. Bars: 25 μm

## 4 DISCUSSION

Malignant gliomas represent one of the most life‐threatening primary brain neoplasms, and the main cause of death for patients is the invasion and metastasis of tumor.^22^ However, while substantial progress to understand the molecular mechanisms of tumor has been made, we still lack enough insight into the mechanisms of the invasion and metastasis in patients with gliomas.

The progress of gliomas is a multistep process involving the balance between tumor suppressor genes and oncogenes. In this study, we found the oncogenicity of 14‐3‐3ζ in the progression of gliomas. The results showed that overexpression of 14‐3‐3ζ was significantly associated with tumor size, recurrence, and weaker DFS rate. In this study, we verified that overexpression of 14‐3‐3ζ promoted gliomas cells proliferation, cell migration, and invasion, which indicated that 14‐3‐3ζ had strong tumorigenicity in gliomas. Our results are consistent with previous reports, which demonstrated that 14‐3‐3ζ overexpression was associated with the cascade of the malignant progression of gliomas.^23^ Unfortunately, the molecular mechanisms of 14‐3‐3ζ underlying invasion remain elusive. According to the results of this study, we present that the oncogenicity of 14‐3‐3ζ dates, at least in part, from the role in promoting the activity of Snail. Snail is a vital inducer of EMT, and the overexpression of Snail correlates with tumor grade and metastasis and predicts a poor outcome with patients for various cancers.^24^ In gliomas cells, it has been reported that Snail could control the differentiation status of gliomas‐initiating cells by regulating BMP and TGF‐β pathways.^25^ These reports are consistent with our data, which proved that 14‐3‐3ζ overexpression promotes the migration and invasion of the gliomas cells.

The article "14‐3‐3ζ promotes gliomas cells invasion by regulating Snail through the PI3K/AKT signaling" was retracted in 2023. Reasons: errors in the data; errors in the images; duplicated images; unreliable results or conclusions.

Our study further indicated that 14‐3‐3ζ promoted the migration and invasion of gliomas cells by regulating Snail via activation of the PI3K/AKT signaling pathway. Previous studies have proved that activation of PI3K/AKT is able to increase the protein expression of Snail, subsequently promoting hepatocellular carcinoma (HCC) cells migration and invasion.^26^ Our data showed that PI3K/AKT was activated when 14‐3‐3ζ was overexpressed, and PI3K/AKT signaling inhibitors markedly attenuated the Snail expression triggered by 14‐3‐3ζ overexpression. These results indicate that 14‐3‐3ζ promotes Snail expression through the activation of the PI3K/AKT signaling pathway. Based on our results and pervious reports, we present a model for how 14‐3‐3ζ promotes gliomas cells invasion.

In conclusion, our data indicated that the 14‐3‐3ζ promotes the migration and invasion of the gliomas cells by regulating Snail through activating PI3K/AKT signaling, and it may act as a potential therapeutic target.

## CONFLICT OF INTEREST

The authors declare no conflict of interest.

## ETHICS APPROVAL AND CONSENT TO PARTICIPATE

The use of human tissues was approved by the Human Research Committee of Huazhong University of Science and Technology (IORG No: IORG0003571). Written informed consent was obtained from each patient. All animal experiments were performed according to the guidelines of care and use of laboratory animals and were approved by the Tongji Medical College Animal Experiments Committee (S777).
